The article "Genome Assembly and Analyses of the Macrofungus Macrocybe gigantea" was retracted in 2024. Reasons: signs of a paper mill; suspected computer-generated content; unreliable results or conclusions; concerns about the data.

# Genome Assembly and Analyses of the Macrofungus *Macrocybe gigantea*

**DOI:** 10.1155/2021/6656365

**Published:** 2021-01-18

**Authors:** Ling Kui, Zhe Zhang, Yangzi Wang, Yesheng Zhang, Shiming Li, Xiao Dong, Qiuju Xia, Jun Sheng, Jian Wang, Yang Dong

**Affiliations:** ^1^College of Biological Big Data, Yunnan Agricultural University, Kunming 650201, China; ^2^School of Pharmacy, Jiangsu University, Zhenjiang 212013, China; ^3^BGI-Shenzhen, Shenzhen 518083, China; ^4^BGI Institute of Applied Agriculture, BGI-Shenzhen, Shenzhen 518120, China; ^5^BGI Education Center, University of Chinese Academy of Sciences, Shenzhen 518083, China; ^6^Yunnan Plateau Characteristic Agricultural Industry Research Institute, Kunming, 650201 Yunnan, China; ^7^Key Laboratory of Puer Tea Science, Ministry of Education, Yunnan Agricultural University, Kunming, 650201 Yunnan, China; ^8^Guangxi Key Laboratory of Medicinal Resources Protection and Genetic Improvement, Guangxi Botanical Garden of Medicinal Plants, Nanning 530023, China; ^9^State Key Laboratory for Conservation and Utilization of Bio-Resources in Yunnan, Yunnan Agricultural University, Kunming 650201, China

## Abstract

*Macrocybe gigantea* (*M. gigantea*) is a macrofungus genus that contains a big number of fairly fleshy gilled mushrooms with white spores. This macrofungus produces diverse bioactive compounds, antioxidants, and water-soluble polysaccharides. However, the genomic resources of this species remain unknown. Here, we assembled the genome of *M. gigantea* (41.23 Mb) into 336 scaffolds with a N50 size of 374,455 bp and compared it with the genomes of eleven other macrofungi. Comparative genomics study confirmed that *M. gigantea* belonged to the *Macrocybe* genus, a stand-alone genus different from the *Tricholoma* genus. In addition, we found that glycosyl hydrolase family 28 (GH28) in *M. gigantea* shared conserved motifs that were significantly different from their counterparts in *Tricholoma*. The genomic resource uncovered by this study will enhance our understanding of fungi biology, especially the differences in their growth rates and energy metabolism.

## 1. Introduction

*Macrocybe gigantea* (*M. gigantea*), which is commonly named *Tricholoma giganteum*, belongs to a genus of fungi in the family of *Tricholomataceae*. *Macrocybe* fungi are widely distributed in tropical regions worldwide, and this genus is related to the genus *Calocybe* [1]. Since the end of the last century, *Macrocybe* has been treated under *Tricholoma* [2]. Pegler et al. separated *Macrocybe* out from *Tricholoma* and ranked it as a stand-alone genus according to morphological and molecular evidence. Previously, most studies of *M. gigantea* were focused on the analysis of antibacterial activities of bioactive compounds, antioxidants, and water-soluble polysaccharides [3–6]. Generally, a single cluster weighs about 20 to 30 kilograms. The largest cluster of giant chanterelles, which was found very recently in Pu'er City of Yunnan Province in China, weighs about 150 kilograms.

The article "Genome Assembly and Analyses of the Macrofungus Macrocybe gigantea" was retracted in 2024. Reasons: signs of a paper mill; suspected computer-generated content; unreliable results or conclusions; concerns about the data.

Due to the lack of a reference genome, most of the macrofungi cannot be studied in the laboratory. However, the rapid development of sequencing methods and analytic tools, which is extensively utilized for the study of evolution, pathology, and molecular population genetics, has been promoting the generation, release, and update of draft data. Recently, several macrofungi genomes have been published, and a lot of large fungal genome projects are in progress [7]. Especially, the Human Microbiome Project [8], the microbial dark matter project, and the 1000 fungal genomes project (http://1000.fungalgenomes.org) [9] have given rise to thousands of microbial genome assemblies; more unprecedented findings are on the way in the short future. In 2018, we reported about 90 draft genome assemblies from different funguses, so far, which is the largest genomic dataset for macrofungi species [7]. As a typical representative of macrofungi, there are a lot of evolutionary and genetic problems to be explored in *M. gigantea*; however, the genome of this species has not been reported.

In this study, the genome of *M. gigantea* was sequenced, and a comparative genomics approach has been used to study it. The results show that different from the *Tricholoma* genus, *M. gigantea* belongs to the *Macrocybe* genus, which is a stand-alone genus. Furthermore, we found that glycosyl hydrolase family 28 (GH28) in *M. gigantea* shared conserved motifs that were significantly different from their counterparts in *Tricholoma*. The genomic data obtained in this study could be a useful resource for the investigation of these macrofungi in the future.

## 2. Materials and Methods

### 2.1. Sequencing and Assembly of the Contig-Level Genome

Sequencing libraries were prepared according to the standard protocol from Pacific Biosciences of California, Inc., and sequenced on the PacBio RS II platform with the P6 polymerase/C4 chemistry (Pacific Biosciences, USA). Then, about 8.7 Gb sequencing data (two times), including 1,135,758 reads, were produced, and the average read length is 7,707 bp (Table 1). We first made corrections on those reads by using the error correction module embedded in Canu (http://canu.readthedocs.org) with a parameter-corrected error rate of 0.045 as the error rate of PacBio reads (15~20%) is high. Subsequently, the corrected PacBio subreads were imported to do genome assembly with Canu [10]. After aligning to the downloaded sequences from GenBank withlength > 1 Kbwith BWA, the contaminant contigs derived from other fungi, bacteria, or human genome were removed.

The article "Genome Assembly and Analyses of the Macrofungus Macrocybe gigantea" was retracted in 2024. Reasons: signs of a paper mill; suspected computer-generated content; unreliable results or conclusions; concerns about the data.

### 2.2. Annotate Tandem Repeats

Genome-wide tandem repeats (TEs) were identified by making use of the Tandem Repeats Finder program with the default settings [11]. A combination of homology-based and *de novo* approaches were used to define the TEs in the *M. gigantea* genome. In the field of homology-based prediction, *RepeatMasker* [12] was implemented to identify TEs against Repbase (Release 16.10; http://www.girinst.org/repbase/index.html) at the DNA level with the default settings. Besides, *Repeat Protein Mask* with the default settings was carried out to identify TEs via the RMBLAST search against the TE protein database at the protein level. For the *de novo* prediction, *Repeat Modeler* (http://repeatmasker.org/) [12] and *LTR FINDER* [13] were utilized to define the *de novo* evolved repeats from the above-assembled genome. Identification of the S-locus TEs in *M. gigantea* and *A. thaliana* was accomplished by the widely used *CENSOR* (http://www.girinst.org/censor/) with the default settings.

### 2.3. Predict Protein-Coding Genes

Both of the *de novo* and homology-based prediction methods were used here to annotate protein-coding genes in the *M. gigantea* genome. All of the coding sequences in the genes of *Laccaria bicolor* Orton, *T. matsutake*, and *Hypsizygus marmoreus* were captured by running the *Phytozome* v9.1 program (http://www.phytozome.net/) and then imported to the homology-based gene annotation process. Subsequently, *TBLASTN* was performed to map the protein-coding sequences of the aforementioned species to the *M. gigantea* genome with the *e*-5 *E*-value and -*F* parameters. For each individual protein, all matched DNA sequences in the reference *M. gigantea* genome were concatenated by *Solar* after filtering the low-quality records. A long protein-coding region was packaged by extending a 2,000 bp fragment at both the upstream and downstream of the concatenated sequence. After that, *GeneWise* [14] was used to predict gene structures one by one with the “new” protein-coding regions. Two *de novo* prediction programs, *AUGUSTUS* [15] and *Genemarker*, were successively used to annotate the protein-coding genes. The protein-coding gene sets in *M. gigantea* predicted by *de novo* and homology-based methods were merged to form a comprehensive and nonredundant reference gene list using *EVidenceModeler* [16]. Again, all programs above were executed with the default settings unless independent indications were given.

The article "Genome Assembly and Analyses of the Macrofungus Macrocybe gigantea" was retracted in 2024. Reasons: signs of a paper mill; suspected computer-generated content; unreliable results or conclusions; concerns about the data.

### 2.4. Gene Family Cluster

All of the coding sequences in the protein-coding genes in *A. ostoyae* C18/9, *P. eryngii*, *C. cinerea*, *C. gibba*, *L. nuda*, *T. matsutake* 945 v3.0, *T. saponaceum*, *T. sp*, *T. terreum*, *T. flavovirens*, *T. bakamatsutake*, and *M. gigantea* were downloaded from JGI Genome Portal and National Center for Biotechnology Information (NCBI). In order to define the gene family clusters among the above species and *M. gigantea*, all-versus-all protein searches using BLASTP with the parameter of “*E* value = 1e^−5^” were performed. Then, OrthoMCL (version 1.4, 17) was employed to handle the high-scoring segment pairs. The MCL package in OrthoMCL was then used to dig the final paralogous and orthologous genes with the ^“^ − abc − I = 1.5” parameter. The result was summarized and shown in the Venn diagram format via a web tool named *VENNY* 2.1 (http://bioinfogp.cnb.csic.es/tools/venny/index.html).

### 2.5. Construct Preliminary Internal Transcribed Spacer Tree

In our database, the sequences of Internal Transcribed Spacers (ITS) were acquired from GenBank following the fungal taxonomic tree, the Catalogue of Life, the Dictionary of Fungi, and its index. The ribosomal DNA, especially ITS1, ITS2, and 5.8S parts of rDNA, was obtained from NCBI and our assembly result. With reference to the classification results of JGI, we selected nearly 300 species of the *Agaricales* to be aligned on NCBI and finally obtained 2,127 of ITS sequences for preliminary classification of *M. gigantea* (Figure 1, Supplemental Table 3). The ITS sequence data were initially aligned by the release of Molecular Evolutionary Genetics Analysis version 5 (MEGA v5.05) with the default settings [17]. Then, the aligned results were manually adjusted. In addition, the Maximum Composite Likelihood analyses were also completed by MEGA with the General Time Reversible plus the Gamma distribution substitution model, aliased as GTR+G. In order to assess the statistical support of clades, 1,000 fast-bootstrap (BS) replications were run. Besides, three species of *Agaricales* affiliated to three different families were selected as the outgroup taxa. The details can be found in Supplemental Table 8.

Because of the numerous insertions and deletions, all of the ITS sequences used in this study cannot be aligned unambiguously. However, in order to get a better and prior understanding of clade diversity within *Agaricus*, the ITS analyses for these sequences were conducted by making use of the Maximum Composite Likelihood (ML) model from various alignment methods [17]. This preliminary ML tree served as a map for sampling strategies, both for sequencing other genes and for the divergence time analysis. 342 samples representing species from each of the recognized sections and main lineages within each section were subsequently selected for generating ITS clade sequence data. Subsequently, the alignments were visually checked and corrected for the striking misaligned positions by MEGA5.05 to maximize primary sequence homology.

The article "Genome Assembly and Analyses of the Macrofungus Macrocybe gigantea" was retracted in 2024. Reasons: signs of a paper mill; suspected computer-generated content; unreliable results or conclusions; concerns about the data.

### 2.6. Additional ITS Analysis with *M. gigantea*

Our focus is to figure out which genus *M. gigantea* belongs to. To this end, we had performed an independent analysis of ITS sequences to identify the “proxy” specimens which can represent them in the multigene phylogeny (Supplemental Table 4). First, the ITS sequence data were aligned by MEGA with the default settings followed by manual adjustments [17]. Then, the maximum-likelihood analyses were performed with the GTR+G substitution model. For the purpose of assessing the statistical support of clades, we had run 1,000 fast-bootstrap (BS) replications under the General Time Reversible model. To get the best DNA models in MEGA5.05, the rates and patterns were filtered from gamma distributed with invariant sites (G+I) by running the program. The ITS sequences were also obtained from NCBI and our above assembly result. All the 553 ITS belonged to nearly 100 species. In fact, we performed BLAST on each species through NCBI and then selected the best 10 of the 50 results to represent the species. We selected the ITS sequences of all the species that can be found in the *Tricholomataceae* and used the same method for phylogenetic analysis. 94 species from *Tricholoma*, 3 species from *Macrocybe*, and *P. eryngii* and *C. cinerea* as outer groups were used in our tree (Supplemental Table 5 and Supplemental Figure2).

### 2.7. Construct Phylogenetic Tree and Estimate Divergence Time

In total, 157 single-copy orthologous genes from the aforementioned species were identified in the gene family cluster analysis. These genes were then imported to construct a phylogenetic tree. Here, for each gene, multiple sequence alignments were performed by employing the *MUSCLE* v.3.7 program with the default settings (http://www.drive5.com/muscle) [18]. For each species, four-fold degenerate sites were extracted from each gene and concatenated into a “supergene.” The *MrBayes* v3.1.2 program (http://mrbayes.sourceforge.net) [18] was utilized to reconstruct the phylogenetic trees among the species.

The *MCMCTREE* program of the *PAML* package [13] was applied here to evaluate the divergence time of *A. ostoyae C18/9*, *P. eryngii*, *C. cinerea*, *C. gibba*, *L. nuda*, *T. matsutake 945 v3.0*, *T. saponaceum*, *Tricholoma_sp_MG77*, *T. terreum*, *T. flavovirens*, *T. bakamatsutake*, and *M. gigantea*. The HKY85 model and the independent rate molecular clock were set to 4 and 2 for computation. The MCMC process in this program was executed 1,000,000 times within the samples, in one of which the frequency was set to 2 after a burn-in of 200,000.

The article "Genome Assembly and Analyses of the Macrofungus Macrocybe gigantea" was retracted in 2024. Reasons: signs of a paper mill; suspected computer-generated content; unreliable results or conclusions; concerns about the data.

### 2.8. Identify Gene Families in *Tricholomaceae*

We obtained *M. gigantea* sequences from the above assembly result. The BLAST program with the *E* value = *e*^−5^ parameter was locally performed with the Hidden Markov Model (HMM) profile in the Pfam database (http://pfam.janelia.org/search/sequence) to capture the candidate gene sequences. Candidate genes containing the known conserved domains were retained, and their presence was checked in the Pfam, SMART (http://smart.embl-heidelberg.de/), and NCBI Conserved Domain (http://www.ncbi.nlm.nih.gov/- Structure/cdd/wrpsb.cgi) databases. The *A. ostoyae*, *P. eryngii*, *C. cinerea*, *C. gibba*, and *L. nuda* sequences were downloaded from the Department of Energy (DOE) in the Joint Genome Institute (JGI) located in America (https://jgi.doe.gov), and the *Tricholomaceae* genome annotation results were downloaded from NCBI.

### 2.9. Detect Contraction and Expansion of Gene Families

*CAFÉ* v2.1 was employed to analyze the evolution of the gene family size according to the stochastic birth and death model [13, 19]. With the divergence time and the calculated phylogeny in hand, *CAFÉ* with the parameters “*p* value =0.05, number of threads = 10, number of random = 1,000, and search for lambda” was used to define the gene families which had experienced the contraction and/or expansion in the aforementioned species.

### 2.10. Detect Positively Selected Genes

In order to screen out the genes under positive selection, we, respectively, blasted the CDS libraries of *C. gibba* and *A. ostoyae C18/9* to the CDS library of *M. gigantea* with the BLASTn program. The best hits were carefully checked by the *Ka/KS Calculator* v.2.0 with the default parameters [19].

Moreover, another approach based upon syntenic comparison was also carried out to define the positively selected genes in *M. gigantea*. Briefly, protein sequences were aligned to themselves by using the BLASTp program. The five alignments at the top for each gene were retained. Then, the high-confidence collinear blocks with the *E* values less than *e*^−10^, and the scores more than 300 were selected by *MCScanX* [20]. For the paired genes inferred from the syntenic alignment, we aligned the protein sequences by using the *CLUSTALW* program [21] and used the result to guide coding-sequence alignments by *PAL2NAL* [21]. In the yn00 program of the PAML package, the Ks and Ka values were calculated using the Yang–Nielson method [13]. A Python script can be run to construct a pipeline including all the calculations. It is available at http://github.com/tanghaibao/biopipeline/tree/master/synonymous_calculation for free download. Again, all programs above were executed with the default settings unless independent indications were given.

The article "Genome Assembly and Analyses of the Macrofungus Macrocybe gigantea" was retracted in 2024. Reasons: signs of a paper mill; suspected computer-generated content; unreliable results or conclusions; concerns about the data.

### 2.11. Parse Gene Structure, Conserved Motif, and Promoter Cis-Acting Regulatory Element

The motif-based sequence analysis tools (*MEME*) suite (http://meme-suite.org/index.html) and TBtools software [22] were used to define the conserved motifs with the following parameters: the number of repetitions is arbitrary, the optimal width of the motif is between 6 and 200 residues, and the maximum number of patterns is 20.

## 3. Results

### 3.1. Genome Assembly of *M. gigantea*

The *M. gigantea* genome was deeply sequenced with the PacBio RSII and PacBio Sequel platforms, which yielded ~8.75 Gb of raw data (213× coverage), totaling 1,135,758 reads (Supplemental Table 1). Ultimately, the sequencing data were assembled with CANU into 336 scaffolds (Table 1). The assembly size was 41.23 Mb, which was smaller than that of *Tricholoma matsutake* (189 Mb), *Tricholoma bakamatsutake* (140.67 Mb), and *Lepista nuda* (44.13 Mb; Supplemental Table 2). The final N50 size was 374,455 bp, and the N90 size was 38,255 bp. The completeness of the genome assembly was evaluated by the Benchmarking Universal Single-Copy Orthologs (BUSCO) analysis, and the result showed that 89.6% of complete BUSCO fungal set genes (*n* = 290) and 6.9% of fragmented BUSCO genes could be found in the *M. gigantea* genome.

In the structural annotation procedure, the genome size of *M. gigantea* was computed as 41.23 Mb, and the number of annotated genes was 11,722. The number was less than the average number among the order *Agaricales*. For instance, *Tricholoma bakamatsutake*, *Coprinopsis cinerea*, and *Lepista nuda* genomes had 14,636, 13,393, and 14,880 predicted genes in their genomes, respectively [7, 23, 24].

In the next step, the OrthoMCL [25] software was used to construct the orthologous groups (OGs) with the best protein models from *Armillaria ostoyae* C18/9, *Pleurotus eryngii*, *C. cinerea*, *Clitocybe gibba*, *L. nuda*, *T.* matsutake 945 v3.0, *Tricholoma saponaceum*, *Tricholoma* sp. MG77, *Tricholoma terreum*, *Tricholoma flavovirens*, *T. bakamatsutake*, and *M. gigantea* [7] with a scalable method. Each constructed OG was a set of proteins and across at least one species. Besides, all of the proteins exist in the 11 listed genomes which represent putative orthologs. The threshold value for all-versus-all BLASTP was set to 10^−8^.

The article "Genome Assembly and Analyses of the Macrofungus Macrocybe gigantea" was retracted in 2024. Reasons: signs of a paper mill; suspected computer-generated content; unreliable results or conclusions; concerns about the data.

Then, gene annotation was carried out based on the OG result. According to the bioinformatics initiative Gene Ontology, all of the 15,788 OGs were imported as a seed for the functional annotation process [26] (Table 1).

### 3.2. Preliminary ITS Tree

In order to understand the evolutionary relationship of *M. gigantea* within clades in *Agaricomycetes*, we performed neighbor-joining bootstrapping (NJ) analyses of the ITS sequence data [27, 28]. We first selected 342 taxa from a total of 2,127 *Agaricomycetes* samples for analyses based on this preliminary NJ tree, after excluding the ambiguous regions (Figure 1). After this, the best scoring ML trees with 342 sequences representing *Agaricomycetes* and bootstrap supported by GTR+G support were shown in Supplemental Figure 1 and Supplemental Table 3. In this tree, the genus *Tricholoma* and *Macrocybe* were clearly divided into two separate branches. The representatives of *Tricholoma*, *T. matsutake*, *T. bakamatsutake*, *T. terreum*, *T. saponaceum*, and *T. flavovirens* were grouped together, and the genus *Macrocybe* and *M. gigantea* were also grouped together. Evidently, *Tricholoma giganteum* was on the branch with the genus *Macrocybe*. In a previous research, Pegler et al. [1, 2, 29] took *T. giganteum* out of *Tricholoma* and grouped it into *Macrocybe*, and our phylogenetic tree supported this conclusion. Both *L. nuda* and *T. matsutake* belonged to the genus *Tricholoma* (http://www.catalogueoflife.org).

To further determine whether *M. gigantea* belonged to the genus *Tricholoma* or *Macrocybe*, we used the previous method (Supplemental Table 4) to select 553 sequences from the *Tricholoma* genus (a total of 369 species, 94 of which had sequence records) and *Macrocybe* genus (a total of 7 members, found that there are 3 members with sequence records) on the Catalogue of Life (Supplemental Table 5), while we also selected *C. cinerea*, *Agaricus parasubrutilescens*, and *P. eryngii* as representatives of another genus in *Tricholomataceae* and select *A. ostoyae* as the outgroup (Supplemental Figure 2). Finally, 90 sequences were selected from the above sequence (Figure 2(a), Supplemental Table 5, 6).

In this multigene tree (Figure 2(a)), three major clades were formed: *Macrocybe*, *Tricholoma*, and outgroup. The *Macrocybe* and *Tricholoma* clades were sister clades to each other, and all collections of *Macrocybe* showed a monophyletic relationship. Sections *Tricholoma* split into multiple clades (orange block). Section *Macrocybe* (light coral block), which contained the species *M. gigantea*, was not strongly supported as a monophyly with 1,000 Bootstrap Replications, but the topological structure of the classification of major species was supported in Zhao's article [28]. One striking exception, however, in this study is some species of the *Tricholoma* were split into another subgenus (e.g., MF034302.1 *Tricholoma sulphurescens*, LT0001741 *Tricholoma inamoenum*, AY462030.1 *Tricholoma bufonium*). We also found that the species named *Tricholoma giganteum* was also clustered on the branch *Macrocybe*, which is consistent with the results of previous scholars [1]. We also obtained the same conclusion that *Tricholoma* and *Macrocybe* were not the same clade by constructing a phylogenetic tree using CDS sequences (Figure 2(d)) [30].

The article "Genome Assembly and Analyses of the Macrofungus Macrocybe gigantea" was retracted in 2024. Reasons: signs of a paper mill; suspected computer-generated content; unreliable results or conclusions; concerns about the data.

### 3.3. Phylogenetic Analysis of *M. gigantea*

The phylogenetic position of many species in the genus *Tricholoma* remains highly contentious [31, 32]. Since the time divergence can be served as a more objective and biologically informative criterion for the delimitation of taxonomic ranks [33], here, we presented a case study in which this criterion was applied for the systematics revision of a fungal genus. As a result, the taxonomic ranks were minimally disrupted as they were recognized in other studies. The uncertainties and limitations of the molecular divergence time estimation had been discussed in van Tuinen and Torres [34].

Phylogenomic analysis based on 1,976 concatenated conserved single-copy genes confirmed the position of *Macrocybe* in the *Tricholomaceae*, with *Pleurotus*, *Armillaria*, and *Coprinopsis* as their outgroup species (Figures 2(a) and 2(d)). We estimated the age of the most recent common ancestor (MRCA) of *Macrocybe* at 125 million years (Myr) and the divergence from *Clitocybe* at 143.5 *Myr* in the Early Cretaceous, which corresponded to the time when the Angiosperms evolved [35].

The genome-wide reconstruction of gene loss and duplication histories in 12 *Agaricales* species recovered an origin for most of the genes, the lineage-specific losses in genus-level groups, and in most of the gene families. 6,630 protein-coding genes were inferred for MRCA of *Agaricales* and 6,417 for the MRCA of *Tricholomaceae* (13 duplications, 186 losses) (Figures 2(b) and 2(c)). Further expansions happened in the 5,546 genes were inferred for the MRCA of *Tricholoma* (60 duplications, 491 losses). Further comparisons of all 12 species revealed 1,237 expanded gene families in the *M. gigantea* genome (Figure 2(c)). Remarkably, the products of many expanded genes even gene families are elements of the degrading enzymes in the plant cell wall (i.e., Cellulase Glyco_hydro_61, hydrophobins, carboxylesterase). The data strongly enhanced the annotated whole-genome sequence of *M. gigantea*.

The article "Genome Assembly and Analyses of the Macrofungus Macrocybe gigantea" was retracted in 2024. Reasons: signs of a paper mill; suspected computer-generated content; unreliable results or conclusions; concerns about the data.

Comparative analysis of *C. cinerea*, *A. ostoyae*, *T. matsutake*, *T. bakamatsutake*, and *M. gigantea* genes defined a total of 17,708 homologous gene families, of which 4,254 gene families were shared by all five species and 476 gene families were *M. gigantea* specific (Figure 2(c)). At the same time, we found that 129 genes were unique to the two species *M. gigantea* and *A. ostoyae*, which have huge fruiting bodies.

### 3.4. Classify Energy Metabolism-Related Genes in *M. gigantea*

The results of Sipos et al. and Peter et al. [36–38] indicated that the pathogenicity mechanisms and the evolution of the unique dispersal of *Armillaria* may have assorted a set of ancestral genetic tools for morphogenesis, complex multicellularity, and wood decay. Therefore, we compared the energy metabolism-related gene composition of *M. gigantea* species to the other *Tricholoma* with diverse lifestyles. Unsurprisingly, *M. gigantea* cause wood rotting like *A. ostoyae* in the saprotrophic phase of their lifecycle, which is reflected in their similar heterotrophic method. The genome has the capability of encoding cellulose-, carboxylesterase-, and glycoside hydrolase, which implies the potential to degrade components of the plant cell wall (Figure 2(d), Supplemental Table 7). *M. gigantea* usually show similar gene counts as *A. ostoyae*, but not so obvious in *Tricholoma*. Besides, some pectinolytic families are overexpressed in *M. gigantea* and *Armillaria*. Pectin-degrading families consist of carbohydrate esterase 8 (CE8), polysaccharide lyase (*PL*)1, PL3 and PL4, *GH28*, *GH88*, and *GH78*. It is worth noting that compared to *Tricholoma*, *GH28*, *PL3*, and *CE8* are significantly enriched in *M. gigantea*. The pectinolytic families of *M. gigantea* are unusual for wood-rotting fungi [39], and they might enable it to quickly gain energy in the wood to avoid competing with other microorganisms.

### 3.5. Identification of the Pectinolytic Families in *M. gigantea*

We focused on *GH28* (*Glyco_hydro_28*) from the pectinolytic families. In sum, 65 candidate gene models related to the *GH28* family of *Pfam* were initially captured. Some erroneously predicted *GH28* gene models were manually removed (i.e., evm. model. tig00000709.146). Finally, according to the presence of apparently complete *GH28* domains, a total of 54 gene models were gathered and annotated as *M. gigantea GH28* genes.

The phylogenetic analysis (Figure 3, Supplemental Table 9) indicated that the *M. gigantea GH28* domains can be separated into four big clades, namely clades I, II, III, and IV [40, 41]. Among these 10 *GH28* proteins, 3 belong to group I, 3 to group II, 2 to group III, and 2 to group IV. The *GH28* members from the phylogenetical species were closely clustered in the same clades. Take the clade IV as an example; it contained the members from *Tricholoma* (*T. matsutake*, *T. saponaceum*, *T. sp.*, *T. terreum*, *T. flavovirens*, *T. bakamatsutake*), which indicates they might be originated from a single ancestral gene or orthologues. Interestingly, three proteins from *M. gigantea* were clustered together with a series of *Armillaria GH28* proteins (in clade I), suggesting that the different evolution patterns of *GH28* in *M. gigantea* and *Armillaria* may occur after their divergence. We also employed the MEME [42] webserver to search the conserved motifs which were shared with the *GH28* proteins. A total of 10 distinct conserved motifs were found. As illustrated in Figures 3 and 4, the 16 members from clade I contained two unique *GH28* domains (Figure 4), indicating potential functional similarities among *GH28* proteins, as only were the motif 5 and the adjacent-motif 7 coexisted in *M. gigantea*, *Armillaria*, and some outgroups *GH28* proteins. The previous study says that the *GH28* family played a major role in the initial stage of the development of fruit bodies [43]. The development of related fruiting bodies requires constant cell division and cell wall disintegration and rereconstruction; the particular motifs might do contribution to the functional divergence of *GH28* genes in a way.

The article "Genome Assembly and Analyses of the Macrofungus Macrocybe gigantea" was retracted in 2024. Reasons: signs of a paper mill; suspected computer-generated content; unreliable results or conclusions; concerns about the data.

## 4. Discussion and Conclusions

The genus *M. gigantea* evolved from saprotrophic ancestors in the *Agaricales*. By comparing the sequences in the genomes of *M. gigantea*, *C. cinerea*, and *A. ostoyae*, we found some specific gene profile similar to *A. ostoyae* in *M. gigantea*. Through the analysis of the genome sequence of *M. gigantea*, we found that *M. gigantea* encode a similar set of PCWDE genes like *A. ostoyae*, but obviously different from *Coprinopsis* and *Tricholoma*.

In previous studies, Singer et al. [44, 45] segregated the large-sized mushrooms of *Tricholoma* into a new sect. Later on, Pegler et al. [1] realized the need to separate this section into a new genus, *Macrocybe*. They also confirmed their hypothesis by molecular analysis using a large subunit (LSU) of rDNA [29, 44]. In the present work, the distinct lineage of *T. giganteum* was reevaluated using protein-coding sequence on the genome [44, 46], and our studies also found that *T. giganteum*, *M. gigantea*, *Macrocybe crassa*, and *M. gigantea* are very close on the branches, they are even divided into the same branch; on the contrary, the branches containing *Tricholoma* and the branches of *Macrocybe* and *M. gigantea* belong to two different sister branches (Figure 2(d)). Mycologists are still hesitant to include their collections in *Macrocybe* [47]; maybe this is a good chance to change it.

The article "Genome Assembly and Analyses of the Macrofungus Macrocybe gigantea" was retracted in 2024. Reasons: signs of a paper mill; suspected computer-generated content; unreliable results or conclusions; concerns about the data.

In our phylogenetic analysis, *M. gigantea* was identified as a *Macrocybe* species and showed significant differences from *Tricholoma*. According to the work of Moncalvo et al. [44], *Macrocybe* is closer to *Entoloma* than *Tricholoma* or *Calocybe*. Perhaps, this is why *M. gigantea* was always assigned to a group far from *Tricholoma* in previous research. The *Tricholomataceae* are a large family of mushrooms within the *Agaricales*. The family is inclusive of any white red or yellow species in the *Agaricales* not already classified as belonging to, e.g., the *Amanitaceae*, *Entolomataceae*, *Hygrophoraceae*, or *Pluteaceae*. We also found similar phenomena when conducting evolutionary analysis, which was that always a few members of the *Tricholoma* genus that will gather into another independent clade. This study provides insights into the distinction between species by comparing differences between genes on the genome. It will further facilitate the understanding of the biology of the *Macrocybe.*

## Figures and Tables

**Figure 1:** Evolutionary relationships of preliminary taxa. The evolutionary history was calculated by the neighbor-joining method. The figure shows an optimal tree with the sum of branch length = 33.54212249. The Maximum Composite Likelihood method was used to compute the evolutionary distances, which generated the units of the number of base substitutions per site. 2,127 nucleotide sequences were involved in this analysis. For each sequence pair, all ambiguous positions were removed.

**Figure 2:** (a) Phylogeny of *Tricholomataceae* generated from Bayesian analysis of ITS sequences, rooted with *A. ostoyae*. Bootstrap support (BS) values > 50% are given at the internode bubbles (BS). We performed the maximum-likelihood (ML) analysis of ITS sequence data by Tamura 3-parameter model (T92)+Gamma Distributed (G) substitution model in MEGA5.05. The clade with a thick branch indicates the part we are interested in. Orange: *Tricholoma*; light coral: *Macrocybe*; cyan: *Agaricus*; khaki: *Pleurotus*; red*: Armillaria*. (b) Parameters of annotated *M. gigantea* genes in comparison with those of the *A. ostoyae*, *P. eryngii*, *C. cinerea*, *C. gibba*, *L. nuda*, *T. matsutake*, *T. saponaceum*, *T.* sp., *T. terreum*, *T. flavovirens*, and *T. bakamatsutake.* (c) Gene family cluster analysis of *M. gigantea*, *A. ostoyae*, *C. cinerea*, *T. matsutake*, and *T. bakamatsutake*. (d) Left panel: Gene family expansion/contraction analysis of *C. cinerea*, *T. bakamatsutake*, *T. matsutake*, *T. flavovirens*, *T. sp.*, *T. saponaceum*, *T. terreum*, *L. nuda*, *C. gibba*, *P. eryngii*, *A. ostoyae*, and *M. gigantea*. Right panel: The right-bottom heat map illustrates the copy numbers of the gene coding plant cell wall degrading enzymes and pathogenicity-related gene families in the 12 species.

The article "Genome Assembly and Analyses of the Macrofungus Macrocybe gigantea" was retracted in 2024. Reasons: signs of a paper mill; suspected computer-generated content; unreliable results or conclusions; concerns about the data.

**Figure 3:** The motif compositions and phylogenetic relationships of *GH28* proteins from 11 different species. (a) An unrooted phylogenetic tree constructed by using the ML method of MEGA. The proteins are clustered into five main clades with a few subclades. The black solid circles indicate *GH28* proteins of *M. gigantea*. Subtree branch lines are colored which indicates different clades. (b) The distribution of conserved motifs in *GH28* proteins. The boxes with various colors stand for the different motifs and their positions in each *GH28* protein sequence.

**Figure 4:** Alignment of multiple *GH28* and selected *GH28* domain amino acid sequences. (a) The basic sequence of all 10 selected motifs. (b), (c) The basic details of motif5 and motif 7.

**Table 1:** Summary of the *M. gigantea* genome assembly features.

Type	Value
Genome size (Mb)	41.23 M
Pair-end libraries	Pacific Biosciences RSII and Sequel
Total reads (#)	1,135,758
Total base (Gb)	8.753(213X)
Genome N50 (kb)	374
Scaffold_reads	336
GC (%)	49.82
Complete Buscos (%)	80.7
Repeat size in genome (%)	9.0338
Gene numbers	11,722

Gene annotation statistics	Value

Total num of genes(glean result)	11,722
Average length gene(bp)	2,019.56
Average no. of cds (bp)	1,544.21
Average no. of exons per gene	6.72
Average exon size (bp)	6.72
Average intron length (bp)	38.23

## Data Availability

The data sets supporting the results of this article are available in NCBI. The raw sequencing reads are available at SRR8617733, and the genome assembly data has been deposited at DDBJ/ENA/GenBank under the accession SJRY00000000. The version described in this paper is version SJRY01000000.

## Supplementary Materials

Supplementary 1 Supplemental Figure 1. Molecular phylogenetic analysis by maximum likelihood method. The phylogeny tree shows the relationships among classes from the phylogenetic analysis of Agaricomycetes and allied phyla computed from the maximum likelihood analysis of ITS sequences data. Bootstrap support (BS) values > 50% are given at the internodes. The thickened branches imply the two types of species we are interested in. The tree with the highest log likelihood (-9,152.4805) is exhibited. The associated taxa were clustered together in the trees, and the percentages are shown close to the branches. Initial tree(s) for the heuristic search were automatically got as follows. When the number of common sites was <100 or less than one-fourth of the total number of sites, the maximum parsimony method was used; otherwise, the BIONJ method with MCL distance matrix was used. A discrete Gamma distribution was employed to model the evolutionary rate differences among sites (5 categories (+*G*, parameter = 0.2228)). The tree is drawn by a scale with the branch lengths measured in the number of substitutions per site. 342 nucleotide sequences were involved in this analysis.

The article "Genome Assembly and Analyses of the Macrofungus Macrocybe gigantea" was retracted in 2024. Reasons: signs of a paper mill; suspected computer-generated content; unreliable results or conclusions; concerns about the data.

Supplementary 2 Supplemental Figure 2. Molecular phylogenetic analysis by maximum likelihood method. The maximum likelihood method was used here to infer the evolutionary history based on the data-specific model. The tree with the highest log likelihood (-9,935.0324) is exhibited. The percentage of trees in which the associated taxa clustered together is shown next to the branches. Initial tree(s) for the heuristic search were obtained automatically as follows. When the number of common sites was <100 or less than one-fourth of the total number of sites, the maximum parsimony method was used; otherwise, BIONJ method with MCL distance matrix was used. A discrete Gamma distribution was used to model evolutionary rate differences among sites (5 categories (+G, parameter = 0.4200)). 553 nucleotide sequences were involved in this analysis.

Supplementary 3 Table S1. The library information and data statistics. This table is a summary of the library, sequence platform, and generated data information.

Supplementary 4 Table S2. The statistics of the fungal genomes used in this paper. WR: wood-rotting; ECM: ectomycorrhizal; LD: litter decomposer; WD: wood decay; SN: saprotrophic nutrition; WR: wood rotting; ECM: ectomycorrhizal; LD: litter decomposer; WD: wood decay; SN: saprotrophic nutrition.

Supplementary 5 Supplemental Table 3. Maximum likelihood fits of 24 different nucleotide substitution models. Note. Models with the lowest BIC scores (Bayesian Information Criterion) are considered to describe the substitution pattern the best. For each model, the AICc value (Akaike Information Criterion, corrected), the maximum likelihood value (lnL), and the number of parameters (including branch lengths) are also presented [1]. Nonuniformity of evolutionary rates among sites may be modeled by using a discrete gamma distribution (+G) with 5 rate categories and by assuming that a certain fraction of sites is evolutionarily invariable (+I). Whenever applicable, estimates of the gamma shape parameter and/or the estimated fraction of invariant sites are shown. Assumed or estimated values of transition/transversion bias (*R*) are shown for each model, as well. They are followed by nucleotide frequencies (*f*) and rates of base substitutions (*r*) for each nucleotide pair. Relative values of instantaneous *r* should be considered when evaluating them. For simplicity, the sum of the *r* values is made equal to 1 for each model. For estimating ML values, a tree topology was automatically computed. The analysis involved 342 nucleotide sequences. Codon positions included were 1st+2nd+3rd+noncoding. All positions with less than 95% site coverage were eliminated. That is, fewer than 5% alignment gaps, missing data, and ambiguous bases were allowed at any position. There were a total of 238 positions in the final dataset. Evolutionary analyses were conducted in MEGA5 [2]. Abbreviations: GTR: General Time Reversible; HKY: Hasegawa-Kishino-Yano; TN93: Tamura-Nei; T92: Tamura 3-parameter; K2: Kimura 2-parameter; JC: Jukes-Cantor. (1) Nei M. and Kumar S. (2000). Molecular Evolution and Phylogenetics. Oxford University Press, New York. (2) Tamura K., Peterson D., Peterson N., Stecher G., Nei M., and Kumar S. (2011). MEGA5: Molecular Evolutionary Genetics Analysis using Maximum Likelihood, Evolutionary Distance, and Maximum Parsimony Methods. Molecular Biology and Evolution (In Press). Disclaimer: Although utmost care has been taken to ensure the correctness of the caption, the caption text is provided “as is” without any warranty of any kind. The authors advise the user to carefully check the caption prior to its use for any purpose and report any errors or problems to the authors immediately (http://www.megasoftware.net). In no event shall the authors and their employers be liable for any damages, including but not limited to special, consequential, or other damages. The authors specifically disclaim all other warranties expressed or implied, including but not limited to the determination of the suitability of this caption text for a specific purpose, use, or application.

The article "Genome Assembly and Analyses of the Macrofungus Macrocybe gigantea" was retracted in 2024. Reasons: signs of a paper mill; suspected computer-generated content; unreliable results or conclusions; concerns about the data.

Supplementary 6 Supplemental Table 4. Maximum likelihood fits of 24 different nucleotide substitution models. NOTE. Models with the lowest BIC scores (Bayesian Information Criterion) are considered to describe the substitution pattern the best. For each model, the AICc value (Akaike Information Criterion, corrected), the maximum likelihood value (lnL), and the number of parameters (including branch lengths) are also presented [1]. Nonuniformity of evolutionary rates among sites may be modeled by using a discrete gamma distribution (+G) with 5 rate categories and by assuming that a certain fraction of sites is evolutionarily invariable (+I). Whenever applicable, estimates of the gamma shape parameter and/or the estimated fraction of invariant sites are shown. Assumed or estimated values of transition/transversion bias (R) are shown for each model, as well. They are followed by nucleotide frequencies (*f*) and rates of base substitutions (*r*) for each nucleotide pair. Relative values of instantaneous *r* should be considered when evaluating them. For simplicity, the sum of *r* values is made equal to 1 for each model. For estimating ML values, a tree topology was automatically computed. The analysis involved 553 nucleotide sequences. Codon positions included were 1st+2nd+3rd+noncoding. All positions with less than 95% site coverage were eliminated. That is, fewer than 5% alignment gaps, missing data, and ambiguous bases were allowed at any position. There were a total of 374 positions in the final dataset. Evolutionary analyses were conducted in MEGA5 [2]. Abbreviations: GTR: General Time Reversible; HKY: Hasegawa-Kishino-Yano; TN93: Tamura-Nei; T92: Tamura 3-parameter; K2: Kimura 2-parameter; JC: Jukes-Cantor. (1) Nei M. and Kumar S. (2000). Molecular Evolution and Phylogenetics. Oxford University Press, New York. (2) Tamura K., Peterson D., Peterson N., Stecher G., Nei M., and Kumar S. (2011). MEGA5: Molecular Evolutionary Genetics Analysis using Maximum Likelihood, Evolutionary Distance, and Maximum Parsimony Methods. Molecular Biology and Evolution (In Press). Disclaimer: Although utmost care has been taken to ensure the correctness of the caption, the caption text is provided “as is” without any warranty of any kind. The authors advise the user to carefully check the caption prior to its use for any purpose and report any errors or problems to the authors immediately (http://www.megasoftware.net). In no event shall the authors and their employers be liable for any damages, including but not limited to special, consequential, or other damages. The authors specifically disclaim all other warranties expressed or implied, including but not limited to the determination of the suitability of this caption text for a specific purpose, use, or application.

Supplementary 7 Supplemental Table 5. Species contained in Tricholoma and Macrocybe from the Catalogue of Life. This table lists 369 living species which belongs to Tricholoma and 6 living species which belongs to Macrocybe, respectively.

Supplementary 8 Supplemental Table 6. Maximum likelihood fits of 24 different nucleotide substitution models. NOTE. Models with the lowest BIC scores (Bayesian Information Criterion) are considered to describe the substitution pattern the best. For each model, the AICc value (Akaike Information Criterion, corrected), the maximum likelihood value (lnL), and the number of parameters (including branch lengths) are also presented [1]. Nonuniformity of evolutionary rates among sites may be modeled by using a discrete gamma distribution (+G) with 5 rate categories and by assuming that a certain fraction of sites is evolutionarily invariable (+I). Whenever applicable, estimates of the gamma shape parameter and/or the estimated fraction of invariant sites are shown. Assumed or estimated values of transition/transversion bias (*R*) are shown for each model, as well. They are followed by nucleotide frequencies (*f*) and rates of base substitutions (*r*) for each nucleotide pair. Relative values of instantaneous *r* should be considered when evaluating them. For simplicity, the sum of *r* values is made equal to 1 for each model. For estimating ML values, a tree topology was automatically computed. The analysis involved 90 nucleotide sequences. The codon positions included were 1st+2nd+3rd+noncoding. All positions with less than 95% site coverage were eliminated. That is, fewer than 5% alignment gaps, missing data, and ambiguous bases were allowed at any position. There were a total of 382 positions in the final dataset. Evolutionary analyses were conducted in MEGA5 [2]. Abbreviations: GTR: General Time Reversible; HKY: Hasegawa-Kishino-Yano; TN93: Tamura-Nei; T92: Tamura 3-parameter; K2: Kimura 2-parameter; JC: Jukes-Cantor. (1) Nei M. and Kumar S. (2000). Molecular Evolution and Phylogenetics. Oxford University Press, New York. (2) Tamura K., Peterson D., Peterson N., Stecher G., Nei M., and Kumar S. (2011). MEGA5: Molecular Evolutionary Genetics Analysis using Maximum Likelihood, Evolutionary Distance, and Maximum Parsimony Methods. Molecular Biology and Evolution (In Press). Disclaimer: Although utmost care has been taken to ensure the correctness of the caption, the caption text is provided “as is” without any warranty of any kind. The authors advise the user to carefully check the caption prior to its use for any purpose and report any errors or problems to the authors immediately (http://www.megasoftware.net). In no event shall the authors and their employers be liable for any damages, including but not limited to special, consequential, or other damages. The authors specifically disclaim all other warranties expressed or implied, including but not limited to the determination of the suitability of this caption text for a specific purpose, use, or application.

The article "Genome Assembly and Analyses of the Macrofungus Macrocybe gigantea" was retracted in 2024. Reasons: signs of a paper mill; suspected computer-generated content; unreliable results or conclusions; concerns about the data.

Supplementary 9 Supplemental Table 7. Species used in comparative genomic analyses. This table lists five main species (chitin, cellulose and hemicellulose, genes implied in pathogenicity, lignin, pectin) and others used in comparative genomic analyses.

Supplementary 10 Supplemental Table 8. Information used for the species originally screened. This table contained the main information which included accession on GenBank, genus, and species used for screening.

Supplementary 11 Supplemental Table 9. Maximum likelihood fits of 54 different amino acid substitution models. Note. Models with the lowest BIC scores (Bayesian Information Criterion) are considered to describe the substitution pattern the best. For each model, the AICc value (Akaike Information Criterion, corrected), the maximum likelihood value (lnL), and the number of parameters (including branch lengths) are also presented [1]. Nonuniformity of evolutionary rates among sites may be modeled by using a discrete gamma distribution (+G) with 5 rate categories and by assuming that a certain fraction of sites is evolutionarily invariable (+I). Whenever applicable, estimates of the gamma shape parameter and/or the estimated fraction of invariant sites are shown. They are followed by amino acid frequencies (*f*) and rates of amino acid substitutions (*r*) for each amino acid pair. Relative values of instantaneous *r* should be considered when evaluating them. For simplicity, the sum of *r* values is made equal to 1 for each model. For estimating ML values, a user-specified topology was used. The analysis involved 54 amino acid sequences. All positions with less than 95% site coverage were eliminated. That is, fewer than 5% alignment gaps, missing data, and ambiguous bases were allowed at any position. There were a total of 56 positions in the final dataset. Evolutionary analyses were conducted in MEGA5 [2]. Abbreviations: GTR: General Time Reversible; JTT: Jones-Taylor-Thornton; rtREV: General Reverse Transcriptase; cpREV: General Reversible Chloroplast; mtREV24: General Reversible Mitochondrial. (1) Nei M. and Kumar S. (2000). Molecular Evolution and Phylogenetics. Oxford University Press, New York. (2) Tamura K., Peterson D., Peterson N., Stecher G., Nei M., and Kumar S. (2011). MEGA5: Molecular Evolutionary Genetics Analysis using Maximum Likelihood, Evolutionary Distance, and Maximum Parsimony Methods. Molecular Biology and Evolution (In Press). Disclaimer: Although utmost care has been taken to ensure the correctness of the caption, the caption text is provided “as is” without any warranty of any kind. The authors advise the user to carefully check the caption prior to its use for any purpose and report any errors or problems to the authors immediately (http://www.megasoftware.net). In no event shall the authors and their employers be liable for any damages, including but not limited to special, consequential, or other damages. The authors specifically disclaim all other warranties expressed or implied, including but not limited to the determination of the suitability of this caption text for a specific purpose, use, or application.
